The article "hERG1 channels modulate integrin signaling to trigger angiogenesis and tumor progression in colorectal cancer" was retracted in 2025. Reasons: errors in the images; errors in the text; duplicated images; unreliable results or conclusions.

# hERG1 channels modulate integrin signaling to trigger angiogenesis and tumor progression in colorectal cancer

**DOI:** 10.1038/srep03308

**Published:** 2013-11-25

**Authors:** Olivia Crociani, Francesca Zanieri, Serena Pillozzi, Elena Lastraioli, Matteo Stefanini, Antonella Fiore, Angelo Fortunato, Massimo D'Amico, Marika Masselli, Emanuele De Lorenzo, Luca Gasparoli, Martina Chiu, Ovidio Bussolati, Andrea Becchetti, Annarosa Arcangeli

**Affiliations:** 1 Department of Experimental and Clinical Medicine, Section of Internal Medicine, University of Florence and Istituto Toscano Tumori (ITT), Florence, Italy; 2 Unit of General Pathology Department of Biomedical, Biotechnological and Translational Sciences (SBiBiT) University of Parma; 3 Department of Biotechnology and Biosciences, University of Milano Bicocca, Milano, Italy

## Abstract

Angiogenesis is a potential target for cancer therapy. We identified a novel signaling pathway that sustains angiogenesis and progression in colorectal cancer (CRC). This pathway is triggered by β_1_ integrin-mediated adhesion and leads to VEGF-A secretion. The effect is modulated by the human ether-à-go-go related gene 1 (hERG1) K^+^ channel. hERG1 recruits and activates PI3K and Akt. This in turn increases the Hypoxia Inducible Factor (HIF)-dependent transcription of VEGF-A and other tumour progression genes. This signaling pathway has novel features in that the integrin- and hERG1-dependent activation of HIF (i) is triggered in normoxia, especially after CRC cells have experienced a hypoxic stage, (ii) involves NF-kB and (iii) is counteracted by an active p53. Blocking hERG1 switches this pathway off also *in vivo*, by inhibiting cell growth, angiogenesis and metastatic spread. This suggests that non-cardiotoxic anti-hERG1 drugs might be a fruitful therapeutic strategy to prevent the failure of anti-VEGF therapy.

The angiogenic switch is a critical step in carcinogenesis^1^,^2^, as is also testified by the clinical application of angiogenesis inhibitors^3^,^4^. Most of the latter achieve their effects by blocking Vascular Endothelial Growth Factor-A [VEGF-A; reviewed in^5^], which has a pivotal role in the angiogenic switch^6^. Accordingly, the first angiogenesis inhibitor to be approved for therapy was the monoclonal anti-VEGF-A antibody bevacizumab^7^. The second generation drugs are instead inhibitors of receptor tyrosine kinase (RTK), which regulate angiogenesis in a less direct way^8^. However, maximizing the efficacy of anti-angiogenic therapy turned out to be more challenging than expected^9^. Differently from what was observed in pre-clinical studies, bevacizumab only improves clinical outcome when combined with chemotherapy, in part because it “normalizes” tumor vessels and improves drug delivery^10^.

However, the greatest therapeutic challenge today is perhaps surmounting the intrinsic tumor resistance to anti-angiogenic drugs and avoiding the rapid re-growth of tumor vessels (with relapse of tumor growth) generally observed on withdrawal from anti-angiogenic treatment^11^. The mechanisms of intrinsic refractoriness as well as acquired resistance to treatment can be partly attributed to the neoplastic cells themselves, which can produce and release alternative angiogenic factors^12^. Moreover, the tumor microenvironment (TM) can promote escape from VEGF-targeted therapy^13^, mainly through the onset of hypoxia^14^. The hypoxic TM stimulates activation of the Hypoxia Inducible Factors [HIFs^13^,^15^,^16^], which in turn up-regulate the transcription of *VEGF-A*^6^,^17^,^18^, as well as of many tumor progression genes^14^. It is worth recalling that in cancer, the expression of HIFs and the subsequent secretion of angiogenic factors can be also abnormally up-regulated under normoxic conditions by different pathways^13^,^19^,^20^, mainly involving Akt and its downstream effectors^21^,^22^. Such process is known as hypoxic mimicry^23^. For example, this can result from mutations of the VHL protein^24^ or from activation of different oncogenes, such as those coding for plasma membrane receptors that regulate the phosphatidyl inositol-3-kinase (PI3K) and hence Akt^25^,^26^,^27^.

The TM also comprises the extracellular matrix (ECM) and its receptors, mainly integrins^28^, which represent “functional hubs”, capable to integrate signals in a bi-directional manner between the TM and the intracellular space of tumor cells (reviewed in^29^). In some cases, integrin function depends on the formation of macromolecular complexes which comprise other membrane receptors, thus constituting signaling platforms at the adhesive sites^30^. An interesting recent development of these studies is the observation that such membrane complexes often include ion channels^31^,^32^. In general, increasing evidence supports the notion that ion channels and transporters control the development of cancer hallmarks in different human cancers^33^,^34^,^35^,^36^. In particular, we previously showed that the K^+^ channels encoded by the human *ether-à-go-go related gene* (K_v_11.1, or hERG1) are often aberrantly expressed in human cancers^37^. In these, hERG1 controls different aspects of the neoplastic cell physiology as it triggers and modulates intracellular signaling cascades^38^ through the assembly of multiprotein membrane complexes which also recruit integrin subunits^39^ and receptors for growth factors^40^ or chemokines^41^. Therefore, hERG1 may be an indispensable component of the “functional hubs” that control tumor angiogenesis^39^,^42^.

Based on these premises we hypothesized that the TM, through the functional interplay between integrins and hERG1, regulates angiogenesis and tumor progression and that this mechanism could contribute to VEGF resistance. Here, we test this hypothesis in CRC cells, because hERG1 is expressed in CRCs^43^ and is a negative prognostic factor in non metastatic patients^44^.

## Results

### β_1_ integrins and hERG1 channels form a functional plasma membrane complex

We first determined whether the physical and functional association between hERG1 and the β_1_ subunit of integrin receptors (hereafter β_1_) found in several tumor cell lines^45^,^46^,^39^ also occurs in CRC cells. Several CRC cell lines were characterized for the expression of β_1_ and hERG1 (Supplementary Table 1 (Table 1S). All of them expressed significant amounts of the β_1_ integrin subunit, but variable levels of functional hERG1 channels. The highest level of hERG1 was observed in HCT116 cells, the lowest in HT29 (Table 1S and Supplementary Fig.1 (Fig. 1S)).

Next, β_1_ was engaged by either cell adhesion onto either fibronectin (FN) or an anti β_1_ activating antibody (TS2/16). Data relative to HCT116 cells seeded onto TS2/16 are reported in Fig. 1A. β_1_ engagement increased the hERG1 current density (Fig. 1A upper panel), reaching average amplitudes of more than 3 pA/pF at −120 mV, after 120 min of incubation. Typical hERG1 currents, measured in HCT116 cells seeded for 120 min onto either TS2/16 or BSA are reported in Fig. 1A, lower panel, along with the stimulation protocol. Full data are in Table 2S. These results are consistent with what was observed in leukemias^46^ and neuroblastomas^45^.

Subsequently, we tested the interaction between hERG1 and β_1_ in CRC cells and found co-immunoprecipitation of the channel protein with β_1_. Assembly of the molecular complex took place in cells cultured in serum (Fig. 1B) and required integrin stimulation by FN (Fig. 1C) or by TS2/16 in suspended cells (Fig. 1D). The complex formation in cells seeded onto FN was reduced by treatment with the hERG1 channel inhibitor E4031 (see Fig. 1E and the analysis in Fig. 1 of Supplementary Densitometric Analysis data (Fig. 1S_DA_)). Hence, both an activated integrin and a functional channel are required for the hERG1/β_1_ complex formation (see the cartoon bottom right in Fig. 1). This indicates that inhibition of the molecular complex can be obtained by targeting either the integrin or the hERG1 channel. Consistent with reports in other cell types^39^, the Focal Adhesion Kinase (FAK) was also recruited into the complex (Fig. 1B).

### The β_1_/hERG1 complex modulates the PI3K-Akt pathway

The signaling pathway downstream to the hERG1/β_1_ complex was analyzed by first determining the role of FAK. FAK was found slightly phosphorylated on tyrosine 397 when associated with hERG1 (Fig. 2S), but was independent of hERG1 activation (i.e. was not affected by E4031; Fig. 2S). This result prompted us to look for signaling proteins other than FAK possibly present in, and activated by, the hERG1/ β_1_ complex.

Our immunoprecipitates always contained the p85 subunit of PI3K (Fig. 2A), which was found to be generally phosphorylated (i.e. activated) in CRC cells (Fig. 2B). Phosphorylated p85 was also recruited by the multi-protein complex (Fig. 2C) and phosphorylation was significantly reduced after addition of either E4031 (Fig. 2B and Fig. 2C) or the B_V_7 β_1_-inhibiting antibody (Fig. 2C). On the contrary, treatment with the β_1_-activating antibody TS2/16 stimulated p85 phosphorylation (Fig. 2C). These results indicate that the p85 subunit of PI3K associates with hERG1 and the β_1_ integrin, to constitute a single macromolecular complex and that its phosphorylation depends on (i) integrin activation and (ii) hERG1 channel activity.

We then studied whether modulation of Akt depended on the above mechanism. Treating CRC cells with either E4031 or B_V_7 decreased Akt activity (Fig. 2D), phosphorylation (Fig. 2E) and nuclear translocation (Fig. 2F). The dependence of Akt activity on the presence of functional hERG1 was further demonstrated by the observation that its activity was considerably lower in HCT116 cells in which hERG1 was stably silenced (HCT116-Sh-hERG1) (characterized for *hERG1* expression in Table 3S), compared to Mock-infected cells (HCT116-PLKO), as well as cells expressing low levels of hERG1 (HT29; Fig. 2D).

Finally, the recruitment of PI3K and Akt in the hERG1/β_1_-dependent pathway (see the cartoon bottom right in Fig. 2) was specific, as the activities of other signaling molecules that are normally activated by integrins, such as the integrin linked kinase (ILK)^41^ and c-Src, were not affected by blocking hERG1 (Fig. 3S).

### Integrin-dependent adhesion and hERG1 activity regulate VEGF-A expression in CRC

We analyzed whether the hERG1/β_1_ complex was functionally involved in tumor angiogenesis, first by determining whether *VEGF-A* expression and VEGF-A secretion depended on integrin and hERG1 activity in CRC cells. The basal levels of secreted VEGF-A, as well as the expression of VEGF-A receptors VEGF-R1 and VEGF-R2, are reported in Table 1S.

*VEGF-A* expression was significantly reduced after addition of B_V_7, whereas it was strongly increased by TS2/16 (Fig. 3A). hERG1 inhibition, obtained applying a mix of three anti-*herg1* (α-*herg1*) siRNAs (whose effects on *hERG1* expression are reported in Table 3S) to HCT116 and HCT8 cells, significantly decreased *VEGF-A* expression, that was constitutively depressed in HCT116-Sh-hERG1 cells (Fig. 3B). Inhibition was also produced by the hERG1 blockers E4031 and Way 123,398 (WAY). Silencing *VEGF-A* through α-*vegf-a* siRNA was taken as positive control (Fig. 3B). Consistently, VEGF-A secretion decreased when hERG1 was inhibited by hERG1 blockers or down-regulated with α-*herg1* siRNAs, as well as in HCT116-Sh-hERG1 cells (Fig. 3C). Once again, the effect of α-*vegf-a* siRNA was taken as control (see the far right bar in Fig. 3C). Blocking hERG1 decreased VEGF-A secretion only in the CRC cell lines that displayed a substantial channel expression (i.e. HCT116 and HCT8), while it was almost ineffective in HT29 cells (Fig. 3C).

These results were further substantiated by overexpressing hERG1 in cells with very low endogenous expression (HEK 293 and HT29). The levels of *hERG1* transcript in transfected cells is reported in Table 4S. Transfection with the *hERG1* cDNA (Fig. 3D, black bar) significantly increased VEGF-A secretion in both cell lines, compared to Mock-transfected cells (Fig. 3D, white bar).

### The β_1_/hERG1/PI3K complex, through Akt, induces HIF(s) transcriptional activation

In cancer cells, *VEGF-A* transcription is regulated by HIFs, both HIF-1 and HIF-2, through O_2_-independent mechanisms, which involve Akt and its downstream effectors (see Introduction). Hence, we first determined that the PI3K/Akt inhibitors LY294002 (LY^47^) and perifosine^48^ decreased VEGF-A secretion (Fig. 3E, left panel). Consistently, silencing either Akt1 or Akt2 strongly reduced the VEGF-A transcript (Fig. 3E, right panel).

Moreover, HIF activity was strongly reduced by PI3K/Akt inhibitors (Fig. 3F). We deepened this point by analyzing the transcription of several HIF-dependent genes after either β_1_ integrin activation or inhibition (by TS2/16 or Bv7, respectively), or hERG1 inhibition (by pharmacological blockade or analyzing HCT116-Sh-hERG1 cells). Both integrin and hERG1 inhibition significantly decreased the transcription of the HIF-dependent genes *GLUT-1*, *LDHA*, and of a specific HIF-2 target, *ANGPTL-4*^17^. Conversely, integrin activation induced an increased expression of all tested genes (Fig. 3G). A significant inhibition of HIF(s)-dependent genes was also observed after silencing Akt1 (Fig. 3G; raw data are in Table 5S). Silencing Akt2 significantly affected only *GLUT-1* transcription level, suggesting a weaker involvement of Akt2 in the above pathway.

Because the effects of silencing Akt and inhibiting hERG1/integrin were not additive, probably these regulators belong to the same signaling pathway, with the integrin and the channel proteins being located upstream (see the cartoon bottom right in Fig. 3).

The β_1_ and hERG1-dependent regulation of HIF transcriptional activity was accompanied by up-regulation of HIF-1α protein (Fig. 4A). We studied whether this depended on either transcription or translation of HIFs. The up-regulation of HIF-1α did not depend on the regulation of HIF protein synthesis by mTORC1 and mTORC2 complex^49^, as neither inhibition or silencing of hERG1 decreased p70S6K or pT37 phosphorylation (Fig. 4B). The transcription of HIF-1α is regulated by the Nuclear Factor-kB (NF-kB)^50^,^51^,^52^,^53^. When HCT116 cells were treated with the NF-kB inhibitor (IKK inhibitor VII), a significant reduction in the expression of *HIF-1α* and *HIF-2α*, as well as of HIF-dependent genes was observed (Fig. 4C, raw data are in Table 5S). Consistently, NF-kB nuclear translocation was enhanced by β_1_ integrin activation as well as inhibited by either blocking the β_1_ integrin or hERG1 or silencing Akt1 (Fig. 4D). On the whole, increased transcription of the *HIF-α* gene(s) seems the main regulatory mechanism sustaining the β_1_ and hERG1-dependent up-regulation of HIF-α(s) in CRC cells. In agreement with this conclusion, we found that the transcription of the two *HIF-* α genes was increased by integrin engagement (Fig. 4E), but decreased by either inhibiting hERG1, blocking β_1_, or silencing Akt1 (Fig. 4F). The outline of the hERG1/β_1_ signaling pathway is in the cartoon bottom right in Fig. 4.

### The β_1_/hERG1/PI3K signaling pathway: relationships with hypoxia and p53

The β_1_/hERG1-triggered signaling pathway identified so far is active in normoxic conditions, a situation rarely observable in tumors, *in vivo*, where hypoxic phases and areas alternate during the natural history of a tumor^54^. We then studied the behavior of such pathway in hypoxia. As expected, the expression of HIF-1α (Fig. 5A) and of HIF-dependent genes increased in hypoxic conditions (Fig. 5B), with a lesser effect on *ANGPTL-4*, in agreement with the observation of 17.

We then mimicked the alternate hypoxic/normoxic conditions which typically occur *in vivo*, either naturally or as a consequence of anti-angiogenesis therapy^11^, **c**ulturing HCT116 cells in hypoxia for 5 hours, and then switching them to normoxia. Cells were seeded either onto BSA or FN and hERG1 was inhibited or silenced. Integrin activation increased *VEGF-A* expression in cells which experienced a hypoxic phase before being switched to normoxia whereas hERG1 inhibition/silencing produced inhibition. The same occurred to the *ANGPTL-4* expression (Fig. 5C) Moreover, the effects were considerably stronger than those observed in cells always maintained in normoxia (Fig. 5C). The same enhancing effect of pre-incubation in hypoxia was observed for *HIF-1α* and *HIF-2α* transcripts (Fig. 5D).

Since a reciprocal influence occurs between hypoxia and p53^55^, we finally investigated whether the integrin- and hERG1-dependent pathway was related to p53 expression and activity. The amount of p53 in HTC116 cells (which express a wild type p53^22^), was increased by integrin activation (TS2), but inhibited by both integrin and hERG1 inhibition (Fig. 5E). In cells not expressing p53 (HCT116 p53^−/−^ cells^56^), the amount of HIF-1α protein increased (Fig. 5F and Fig. 5S_DA_ for densitometric analysis), suggesting an inhibiting role of p53 on HIF-1α, which in turn counteract the activation exerted by the β_1_/hERG1-triggered pathway. According to this hypothesis, the increase of *VEGF-A* expression by FN and its inhibition by hERG1 blocking were more evident in HCT116 p53^−/−^ cells compared to p53 wild type cells (Fig. 5G). The complete hERG1/β_1_-dependent pathway is in the cartoon bottom right in Fig. 5.

### hERG1 channels regulate tumor angiogenesis in vivo

We then determined whether the hERG1-dependent regulation of VEGF-A also occurred *in vivo*, and was relevant to the control of tumor angiogenesis. Notably, the VEGF-A secreted by CRC cells does not have an autocrine effect because these cells lack the main VEGF receptors (Table 1S).

We adopted two different experimental procedures (for details, see Supplementary Information):

#### a) in vivo effects of cells overexpressing or not expressing hERG1

HEK 293 cells overexpressing hERG1 (HEK-hERG1) or HCT116-Sh-hERG1 cells were injected subcutaneously into nu/nu mice. As controls, we used HEK-Mock (see Fig. 3D) and HCT116-PLKO cells (see Fig. 2E). The cell masses produced by injection of HEK-hERG1 cells were positive to VEGF-A staining, while those produced by HEK-Mock were negative (Fig. 4S, panel A). Masses from HEK-hERG1 cells displayed a higher total vascular area per microscopic field (see Supplementary Information), as evaluated by CD34 staining. Similarly, tumor masses produced by injection of HCT116-PLKO cells were positive for VEGF-A staining, while those produced by HCT116-Sh-hERG1 cells only showed a faint VEGF-A signal (Fig. 4S, panel B) and an even lower amount of *VEGF-A* transcript (see Supplementary Information).

Interestingly, masses from HEK-hERG1 cells displayed a higher volume compared to the masses obtained by injection of HEK-Mock cells (Fig. 6A). Consistently hERG1 silencing led to significant decrease of the tumor mass volume (Fig. 6B) and of Ki67 staining (Fig. 4S, panel C). The masses obtained by injection of HCT116-Sh-hERG1 cells maintained the *hERG1* silencing throughout the *in vivo* experiment (see Supplementary Information).

#### b) in vivo treatment with hERG1 blockers

The tumor masses arising from subcutaneous injection of HCT116 cells in nu/nu mice were analyzed after treating mice with the hERG1 blockers. This experimental protocol did not alter the behavior, vitality or electrocardiographic properties of treated mice^41^. Treatment with hERG1 blockers was accompanied by a strong decrease of tumor volume (Fig. 6C), and decreased expression of VEGF-A, pAkt and Ki67 (Fig. 6D). Tumor masses arising in mice treated with hERG1 blockers displayed a strong decrease of the total vascular area per microscopic field (Fig. 6F, graph on the right), accompanied by a higher degree of perivascular fibrosis (see arrows in Fig. 6F), as well as by a decrease of pAkt levels, and a lower HIF-1α expression (Fig. 6E and Fig. 6S_DA_ for densitometric analysis), compared to those in control mice.

The effects of blocking hERG1 were also analyzed in mice injected with HCT116- p53^−/−^ cells, which up-regulate HIF-1α (Fig. 5F). These cells produced bigger subcutaneous masses (Fig. 6C, white squares), with increased angiogenesis (Fig. 6F)^22^. In this case, the inhibitory effect of E4031 on either tumor masses (see the white circles in Fig. 6C) or tumor vessels was even stronger (Fig. 6F).

Next, we studied the effects of hERG1 blockers in an orthotopic CRC murine model, detailed in the Supplementary Information. At the time of death, control mice displayed macroscopic (arrows in Fig. 7A) tumor masses and liver metastases which display the presence of many human MHCI (hMHCI)-positive tumor cells (Fig. 7A, panels on the right marked as “liver staining”). An immunohistochemical signal for hMHCI was also detected in tumor masses and **in** small areas of the coecum (Fig. 7C, CONTROL), in the vicinity of the injection site, which showed no macroscopic tumor mass. Moreover, control mice were characterized by the presence of numerous metastatic foci, as well as by the occurrence of complications such as ascites (Table 1). E4031-treated mice did not show macroscopic tumor masses in the site of CRC cell injection (Fig. 7B), neither the presence of liver metastases, although microscopic hMHCI-positive tumor aggregates (Fig. 7C panels on the right, black arrows) were detected. E4031-treated mice did not show signs of macroscopic local growth or invasion, nor any evidence of distant metastases (Table 1).

Finally, we analyzed the effect of pharmacological block of hERG1 in a liver metastases model, detailed in the Supplementary Information. In this case, E4031 delayed the onset of metastatic disease (Fig. 7D) and significantly decreased the number of macroscopic (Fig. 7E and Table 2) and microscopic (Table 2) liver metastases. Moreover, liver metastatic foci of E4031-treated mice displayed a larger necrotic area (Fig. 7F, upper panels stained with H&E), and a lower VEGF-A staining (Fig. 7F, lower panels and Supplementary Information), compared to the controls.

## Discussion

Most of the angiogenesis inhibitors currently used for cancer treatment achieve their effects by blocking VEGF-A. This stops angiogenesis and destroys part of the tumor vasculature, which leads to a hypoxic state inside the tumor mass. Moreover, the ensuing normalization of the tumor vessels promotes the delivery and hence the efficacy of chemotherapeutic drugs^4^. Nonetheless, although blocking VEGF-A slows the growth of many primary tumors and metastases, most advanced cancer can escape from anti-angiogenesis therapy. Paradoxically, those VEGF-A inhibitors that slow tumor growth can also promote tumor escape and progression^9^. Hence, multiple strategies for preventing escape are under investigation. Full success implies the discovery of alternative mechanisms/signaling pathways that can trigger either the expression of angiogenic factors other than VEGF-A, or otherwise favor tumor invasiveness and metastases^57^. We tested the hypothesis that the TM, through the functional interplay between the ECM and integrin receptors, could activate signaling pathways which regulate angiogenesis and tumor progression, hence putatively bypassing VEGF-A inhibition.

Beyond its canonical role in excitability, hERG1 is emerging as a major regulator of intracellular signaling in tumor cells. This role relies on its ability to assemble with partner proteins, and particularly adhesion receptors of the integrin family^31^. In CRC cells, after β1 engagement hERG1 currents were approximately tripled, thus reaching amplitudes of more than 300 pA (corresponding to average densities of about 3 pA/pF), at −120 mV (Table 2S) in high extracellular K^+^ concentrations ([K^+^]_o_). The steady-state currents at physiological V_rest_ and [K^+^]_o_ would be considerably smaller. However, it should be recalled that the maximal steady-state open probability of hERG1 (the peak of the “window current”) is around −40 mV^58^. Moreover, in the high-resistance tumor cell lines, a few tens of pA are sufficient to produce significant changes in V_rest_^45^,^59^. In addition to the increase in hERG1 currents, β1 activation leads hERG1 to form a macromolecular membrane complex that comprises the β_1_ integrin subunit and the p85 subunit of PI3K. Recruitment of p85 inside the complex has two major consequences: i) it facilitates translocation of PI3K towards its physiological membrane substrates; ii) it determines a hERG1-dependent PI3K phosphorylation, without the need of intermediate cytosolic proteins (e.g. FAK, ILK, Src).

Moreover, inhibition of hERG1 (with channel blockers or RNA interference) decreased VEGF-A secretion. The effect of hERG1 channels on VEGF-A secretion turned out to be mediated by transcriptional regulation of *VEGF-A*, which involves the HIF-1 transcription factor^4^. Collectively, the integrin and hERG1-triggered signaling pathway we have defined affect HIF activity (i) through the involvement of Akt1, ii) through the transcriptional regulation of *HIF-1α* and *HIF-2α*, similarly to what occurs in vascular smooth muscle cells treated with Angiotensin II^60^; (iii) independently from m-TOR. A similar m-TOR independent, Akt-dependent regulation of HIF protein synthesis was reported, in CRC cells, by Pore et al^61^. However, the integrin and hERG1-triggered pathway affects HIF protein synthesis through the activity of NF-kB, which has been reported to be one of the main regulators of HIF transcription in different cellular systems^50^,^51^,^52^,^53^. Moreover, the integrin- and hERG1-dependent upregulation of HIF(s) is apparently counterbalanced by p53. Indeed, it is well known that p53, through MDM2, can degrade HIF proteins and hence inhibits the angiogenic switch^22^. Although the link between NF-kB and p53 is still controversial^62^, it is intriguing to speculate that NF-kB and p53 can be oppositely regulated by Akt, once it is directly activated by PI3K, when the kinase is linked to the β_1_/hERG1 complex, and is activated by cell adhesion.

A further indication that the β_1_/hERG1/PI3K-triggered signaling pathway is relevant for cancer biology is that the modulation of HIF transcriptional activity was stronger on normoxic CRC cells, and even more during recovery from deep hypoxia. The latter mimics not only the hypoxic state that characterizes the initial stages of tumor progression^54^, but also the situation experienced by tumor cells during (and after interruption of) anti-angiogenesis therapy.

These observations have potentially relevant therapeutic consequences. In fact, consistently with the signaling pathway described in CRC cells *in vitro*, we showed that hERG1 activity determines neo-angiogenesis and the growth, invasion and metastatic spread of CRC cells *in vivo*. The effects of hERG1 blockers were more potent when tested on p53^−/−^ cells. In other words, when the p53-centered control of cellular apoptosis and shortage of HIF activity was impaired, the ECM/hERG1-dependent stimulation of HIF activity was stronger. The greater efficacy of hERG1 blockers in p53 loss/mutated CRC may be particularly relevant in oncology, as these tumors usually show a greater chemoresistance.

In conclusion, hERG1 represents a tumor progression gene. This has been recently substantiated by studies on chemically induced CRC and transgenic mouse models^63^. These observations, together with the present data, demonstrate that tumor cells use a peculiar hERG1-centered mechanism to regulate angiogenesis, which can be modulated by using hERG inhibitors^64^. Moreover, we here suggest the possibility that non cardiotoxic hERG1 blockers can be used, in association with anti-VEGF drugs, to prevent or bypass anti-angiogenesis therapy resistance. However, before reaching the clinical setting, it will be necessary to exclude the cardiac side effects of the hERG1 blockers to be included in the therapeutic schedule. To this purpose, in an acute leukemia model we have recently shown that non-cardiotoxic hERG1 blockers, such as macrolide antibiotics, display the same therapeutic effects as the specific, potentially cardiotoxic, hERG1 blockers^41^. These results provide a suggestion on how to proceed to test hERG1-targeted anti-angiogenesis therapy in CRC cancers.

## Methods

### Cell cultures

Colorectal cancer (CRC) cell lines HCT116, HCT8, were cultured in RPMI 1640 (Euroclone; Milan, Italy) with 10% Fetal Calf Serum (FCS) (Euroclone Defined; Euroclone; Milan, Italy). HT29 cells were cultured in McCoy's medium with 10% FCS. HCT116 and HT29 cells were kindly provided by Dr. R. Falcioni (Regina Elena Cancer Insitute, Roma). HEK-Mock and HEK-hERG1 cells were obtained by transfecting HEK 293 cells with the pEGFP-C1 plasmid (Clontech; Mountain View, CA, USA) and with a pEGFP-C1 hERG1 plasmid (the kind gift of Dr. L. Pardo, Max-Planck-Institut für experimentelle Medizin, Göttingen, Germany). Stable transfectants were selected and maintained in DMEM with 10% FCS (Euroclone, Milan, Italy) and Geneticin (800 mg/ml).

### Treatment with hERG1 inhibitors

When hERG1 inhibitors (E4031 or WAY) were added to protein-containing media, they were used at a final concentration of 40 μM, as explained in 42.

### VEGF-A secretion

Cells were seeded into 24-well cell culture plates at 2 × 10^5^ cells/ml in standard culture medium. After twenty-four hours, the medium was removed and 0.5 ml of Optimem (Gibco; Carlsbad CA, USA) was added. After an additional twenty-four -hours incubation, the medium was collected and VEGF-A measured using the DuoSet ELISA Development System (R&D Systems; Wiesbaden, Germany). Cells were recovered and counted to normalize the VEGF-A secretion data. When needed, hERG1-specific inhibitors E4031 or WAY were added along with Optimem, as well as PI3K/Akt pathway inhibitors LY294002 (10 μM, Sigma) or perifosine (20 μM, kindly provided by Dr. A. Martelli, University of Bologna).

### Cell transfection

Transient and stable transfections described in the text were performed using Lipofectamine 2000 reagent (Invitrogen) or Hiperfect Transfection Reagent (Qiagen) for Akt1, Akt2, following the manufacturer's instructions.

For hERG1 stable silencing in HCT116 cells, a commercially available TRC shRNA-library (Open Biosystems) was used. For detailed description see Supplementary Information.

### HIF activity

The hypoxia responsive element-luciferase reporter gene vector was kindly provided by Dr. A Giaccia (Stanford University School of Medicine, Stanford, USA). For detailed description see Supplementary Information.

### RNA extraction, reverse transcription and Real-time Quantitative (RT-qPCR)

RNA extraction, reverse transcription and RT-qPCR were performed as in 40. Further details and the complete list of primer's sequences are reported in Supplementary Information.

### Protein extraction, immunoprecipitation (IP) and western blot (WB)

Total and membrane protein extraction were performed by standard methods using 1× lysis buffer (Cell Signaling Technology). WBs were carried out as described in 43. IP experiments were performed according to 39. For the experiment with the activating monoclonal anti-β1 antibody (TS2/16), cells were resuspended in a solution containing 20 μg/ml of antibody in DMEM + BSA and kept in suspension through continuous low speed stirring for thirty minutes at 37°C. For further details and the complete list of antibodies used see Supplementary Information.

### In vivo experiments using mice models

Each *in vivo* mouse model is extensively described in Supplementary Information.

All experiments on live vertebrates were performed in accordance with relevant guidelines and regulations. We confirm that the Ethical Commitee of the University of Firenze approved all the experiments described in this paper.

### Histological analysis

IHC was performed as reported in 43. Staining with anti-CD34 mouse monoclonal antibody (Cederlane Laboratories, 1:100 dilution) was performed after antigen retrieval was carried out by irradiating the slides in a microwave for twenty minutes at 700 W in citrate buffer (pH 7.8). Images were acquired on a Leica DM 4000B microscope with a Leica DFC 320 camera using Leica QWin software (Leica Microsystems; Milan, Italy).

## Author Contributions

O.C. and F.Z. identified the proteins involved in the hERG1/β_1_ complex and characterized the downstream signaling pathway. O.C. performed the experiments in normoxia and hypoxia conditions. S.P., E.L. and M.S. performed the IHC experiments. S.P., M.S. and O.C. performed the in vivo experiments; AFiore contributed to Western Blot experiments; AFortunato produced and characterized the Sh-hERG1 model and contributed to the characterization of the orthotopic model; M.D. and L.G. performed the patch-clamp experiments; M.M. was enrolled for imaging experiments and analysis. E.D.L. produced the orthotopic model; M.C. and O.B. contributed to unravel the mTOR involvement in the signaling cascade; A.B. supervised the patch-clamp experiments and critically wrote the paper. A.A. designed the research, critically interpreted the data and wrote the paper. All authors reviewed the manuscript.

## Supplementary Material

Supplementary Information Supplementary Information

## Figures and Tables

**Figure 1:** Physical and functional characterization of the hERG1/β_1_/FAK complex in GI cancer. (A) Effects of β_1_ stimulation on hERG1 currents of HCT116 cells seeded on TS2/16 or BSA coating. Left panel: hERG1 current density was measured as described in 45 (see also Table 2S for details). Data are mean ± SEM calculated on the number of cells shown above each experimental point. Time point 0 refers to the time at which cells were seeded on the different substrates. Control means cells seeded in standard conditions (RPMI + 10% FCS) for 120 min. Lower panel: current traces of cells seeded onto BSA (250 μg/ml) and TS2/16 (20 μg/ml) for 120 min. See also Fig.1S to compare hERG1 current traces registered in standard culture conditions. (B) Physical association between hERG1 channels, β_1_ integrin and Focal Adhesion Kinase in CRC cells. (C–D) Effect of cell adhesion onto Fibronectin (FN, 100 μg/ml) (C) or β_1_ stimulation through the activating TS2/16 antibody (20 μg/ml) in cells kept in suspension (D) on β1/hERG1 complex assembly. (E) Effects of the hERG1 blocker E4031 (40 μM) on hERG1/β_1_ complex assembly in cells cultured on FN or BSA. Data were analyzed using ImageJ, and graphs, reported in the Supplementary Information section titled Supplementary Densitometric analysis data (Fig. 1S_DA_), were plotted by Microcal Origin 6.0. Full-length blots are reported in Supplementary Information section titled “Full-length blots relative to the cropped images showed in the main Figures”.

**Figure 2:** The hERG1/β_1_ integrin complex modulates phosphorylation of p85-PI3K and Akt activation. (A) p85 participates in the hERG1/β_1_/FAK complex. (C) p85 is phosphorylated in CRC cell lines, and its phosphorylation is significantly affected by hERG1 blocking. Parallel IP were done using rabbit IgG as negative control. (B–C) The p85 associated with the hERG1/β1 complex is phosphorylated (B), and its phosphorylation is modulated by hERG1 and β1 inhibition or integrin activation (C). (D–E) The effects of the E4031 on Akt activity (D) and on Akt phosphorylation (E) in HCT116, HCT8 and HT29 cell lines, as well as in HCT116 transfected with the pLKO.1 empty vector (HCT116-PLKO) or in hERG1-silenced HCT116 cells (HCT116-Sh-hERG1). Data were analyzed using ImageJ, and graphs, reported in Fig. 2S_DA_ were plotted by Microcal Origin 6.0. (F) Immunofluorescence (IF) staining using an anti-Akt (Santa Cruz, SC-8312, dilution 1:500) on control, E4031 or anti-β1 (Bv7) treated HCT116 cells. Negative control is represented by Akt1/2-silenced cells (e.g. cells transfected with siRNA anti-Akt1 and 2 (see Supplementary Information section Materials and methods)). IF protocol was performed as detailed in Supplementary Information. Nuclear/cytoplasmic staining ratios measured by ImageJ (see Supplementary Materials and methods for further details) were the following: Control = 1.8 ± 0.46, E4031 = 0.18 ± 0.028; anti-β1 Bv7 = 0.24 ± 0.025. ** p < 0.02. Full-length blots are reported in Supplementary Information section titled “Full-length blots relative to the cropped images showed in the main Figures”.

**Figure 3:** Characterization of the β1/hERG1-dependent signaling pathway able to influence VEGF-a expression and secretion in HT116 cells. (A) Effect of β1 inhibition or activation on *VEGF-A* expression. (B) *VEGF-A* expression in HCT116 treated with E4031 or WAY (40 μM), in HCT116 and HCT8 transiently transfected with a mix of α-*herg1* siRNAs 1 + 3 or in HCT116-Sh-hERG1. Controls are represented by cells cultured in standard conditions for the pharmacological treated samples, by HCT116-PLKO cells for HCT116-Sh-hERG1 and by HCT116 transfected with siRNA negative control for siRNAs 1 + 3, respectively. (C) Effect of hERG1 blocking on VEGF-A secretion in HCT116 and HCT8 cells. Cells were also used for RNA extraction and RT-qPCR assay shown in Table 3S. Data are means ± SEM of two-four separate experiments, each carried out in duplicate. (D) VEGF-A secretion in HEK-Mock and HEK-hERG1 cells and in HT29-Mock and HT29-hERG1 cells. For quantitative analysis of hERG1 expression, see Table 4S. (E) Effects of PI3K/Akt inhibitors LY294002 and perifosine on VEGF-A secretion (left panel) and of α-Akt1 and α-Akt2 siRNAs on *VEGF-A* expression (right panel). Data are reported as the percentage of control ± SEM of two experiments, each carried out in triplicate. (F) Effects of PI3K/Akt inhibitors LY294002 and perifosine, on HIF-1 transcriptional activity. Data are means ± SEM of three separate experiments. (G) Fold induction of HIF(s) target genes after hERG1, β1 inhibition and activation or after Akt1/2 silencing. Data are means ± SEM of three separate experiments, each carried out in duplicate. *GLUT1*, glucose transporter 1; *LDHA*, lactate dehydrogenase A; *ANGPTL-4*, angiopoietin-like 4.*: p < 0.05; **: p < 0.02; ***: p < 0.01 (Student's t test). Raw data are in Table 5S.

**Figure 4:** Characterization of the signaling pathway downstream the β1/hERG1/PI3K complex. (A) Effect of pharmacological and biomolecular hERG1 inhibition on HIF-1α protein. (B) Evaluation of the activation of mTOR signaling pathway components (mTORC-1 and 2) in HCT116 treated or not with E4031 (40 μM) as well as in HCT116-PLKO and HCT116-Sh-hERG1 cells. Rapamycin (100 nM) was applied for 3 hours as mTORC-1 internal control. (C–D) The effect of NF-kB inhibition on HIF(s) expression and transcriptional activity. RT-qPCR (C) and IF (D) experiments were performed seeding cells on FN coated dishes (100 μg/ml) for 3 hours, treated or not of the IKK inhibitor VII (1 μM). RT-qPCR data are means ± SEM of two separate experiments, each carried out in duplicate. IF staining on NF-kB p65 subunit performed on control (siRNA negative control, Qiagen), anti-TS2/16, anti-β1 Bv7, E4031 treated HCT116 cells and on HCT116 cells transfected with anti-Akt1 or anti-Akt2 siRNAs after FN seeding. Nuclear/cytoplasmic staining ratios measured by ImageJ (see Supplementary Materials and methods for further details) were the following: siRNA neg = 1.1 ± 0.04; anti-TS2/16 = 1.61 ± 0.2; anti-β1 Bv7 = 0.21 ± 0.092; E4031 = 0.13 ± 0.089; anti-Akt1 = 0.51 ± 0.04; anti-Akt2 = 0.98 ± 0.03. * p < 0.05. (E–F) Effects of integrin activation (E) as well as hERG1, β1 and Akt inhibition (F) on HIF(s) transcription. Data are means ± SEM of three separate experiments, each carried out in duplicate. * p < 0.05; ** p < 0.02; *** p < 0.01 (Student's t test). Raw data are in Table 5S. Full-length blots are reported in Supplementary Information section titled “Full-length blots relative to the cropped images showed in the main Figures”.

**Figure 5:** Role of hypoxia and p53 on the β1/hERG1/PI3K signaling pathway. (A) Effect of hypoxia in HCT116 and HCT8 on HIF-1α protein. (B) Effect of hypoxia on HIF(s) target genes. (C–D) Effect of a cycle of an alternate hypoxic (5 h)/normoxic (4 h) condition, compared to a standard incubation in normoxia (5 h + 4 h) on HIF(s) angiogenic target genes (C) and HIF(s) transcripts (D). (E–F) Study of p53 involvement in the regulation of HIF-1α protein. In the left panel is reported a WB showing the effects of hERG1 and β1 inhibition, as well as β1 activation, on p53 protein. Densitometric analysis data were analyzed using ImageJ, and graphs reported in Fig. 5S_DA_, were plotted by Microcal Origin 6.0. (G) Percentage of E4031 inhibition on WT and p53-/- HCT116 cells cultured in FN. Raw data and Pfaffl analysis are reported in Table 5S. Data are means ± SEM of three separate experiments. * p < 0.05; ** p < 0.02; *** p < 0.01 (Student's t test). Full-length blots are reported in Supplementary Information section titled “Full-length blots relative to the cropped images showed in the main Figures”.

**Figure 6:** Role of hERG1 channels in the regulation of in vivo tumor growth and intratumoral angiogenesis in immunodeficient mice. (A) Volume of tumor masses obtained after injection of HEK-Mock and HEK-hERG1 cells. Data are reported as the mean ± SEM of three tumor masses. (B) The same experiments performed using HCT116-PLKO and HCT116-Sh-hERG1 cells. (C) Time course of tumor growth in control (), WAY- () and E4031 ()-treated mice, as well as untreated () and E4031 ()-treated mice injected with HCT116 p53-/- cells. (F) Histological analysis of VEGF-A, pAkt and Ki67 staining of tumor masses obtained in control and WAY-treated mice after injection of CRC cells. Bar: 100 μm for VEGF, 100 μm for Ki67, 100 μm for pAkt. (E) WB analysis of Akt phosphorylation and HIF expression in tumor masses obtained from the injection of HCT116 cells. For further details regarding densitometric analysis, see Fig. 6S_DA_. (F) CD34 staining of control and E4031-treated mice, as well as untreated and treated mice injected with p53^−/−^. Further descriptions are reported in Supplementary Information. Full-length blots are reported in Supplementary Information section titled “Full-length blots relative to the cropped images showed in the main Figures”.

**Figure 7:** Effects of hERG1 blockers in orthotopic and direct metastasis CRC mouse models. (A–B) Representative macroscopic images of the abdomen of control (A) and E4031-treated (B) mice (IP, 20 mg/Kg). Liver: gross images. Both hematoxylin/eosin (H&E) and hMHCI staining (black arrows) of liver sections (A, Control mice, staining of liver metastases sections; B, E4031-treated mice, staining of liver sections) are reported. (C) IHC experiments on control mice (CONTROL) and E4031-treated (E4031) mice. Both hematoxylin/eosin (H&E) and hMHCI staining of tumor masses and of a site of the coecum without macroscopic tumor masses (CONTROL), and of a site of the coecum without macroscopic tumor masses (E4031-treated)) are reported. Black arrows indicate the anti-hMHC staining. Bar: 100 μM for H&E and for hMHC. (D) Representative pseudo-color BLI images tracking HCT116-luc cells emission in nude mice, 13 days after splenic HCT116-luc injection. Color bar represents light intensity levels reported as counts per minute (cpm). (E) Livers from animals sacrificed three weeks after cell injection and two weeks after beginning the pharmacological treatment. (F) H&E and VEGF-A staining revealing larger necrotic areas and the presence of a higher amount of VEGF-A (brown staining) in Control compared to E4031-treated mice.

**Table 1:** Quantitative evaluation of local tumor growth, invasion, distant metastases and complications in control and E4031-treated mice (20 mg/Kg). (+++ = high number of neoplastic masses, ++ = several neoplastic masses, + = few neoplastic masses)

ORTOTHOPIC MODEL		
Local tumor growth	Control	E4031
Coecum	**+++**	**-**
**Invasion**		
Intestin	**++**	**-**
**Metastasis**		
Peritoneum	**++**	**-**
Diaphragm	**+++**	**-**
Liver	**++**	**-**
Spleen	**++**	**-**
Kidneys	**+**	**-**
**Complications**		
Ascites	**++**	**-**

**Table 2:** Number of hepatic macroscopic and microscopic lesions as well as % of necrotic area of livers reported in Fig. 7E–F. Further descriptions are reported in Supplementary Information

LIVER METASTASES MODEL		
Metastases	Control	E4031
Macroscopic metastases	**19.3 ± 3.50**	**9.85 ± 4.80**
Microscopic metastases (number/microscopic field)	**4.0 ± 0.70**	**1.2 ± 0.14**
% necrotic area/total metastases area	**2.1 ± 0.30**	**8.55 ± 0.36**
